This article has been retracted.

# Dual targeting of RANKL and PD‐1 with a bispecific antibody improves anti‐tumor immunity

**DOI:** 10.1002/cti2.1081

**Published:** 2019-09-27

**Authors:** William C. Dougall, Amelia Roman Aguilera, Mark J. Smyth

**Affiliations:** ^1^ Immunology in Cancer and Infection Laboratory QIMR Berghofer Medical Research Institute Herston Qld Australia

**Keywords:** bispecific antibody, metastasis, PD‐1, RANKL, TNFSF11, tumor immunity

## Abstract

**Objectives:**

The addition of RANKL/RANK blockade to immune checkpoint inhibitors (ICIs) such as anti‐PD‐1/PD‐L1 and anti‐CTLA4 antibodies is associated with increased anti‐tumor immunity in mice. Recent retrospective clinical studies in patients with advanced melanoma and lung cancer suggest the addition of anti‐RANKL antibody to ICI increases the overall response rate relative to ICI treatment alone. Based on this rationale, we developed a novel bispecific antibody (BsAb) co‐targeting RANKL and PD‐1.

**Methods:**

We characterized target binding and functional activity of the anti‐RANKL/PD‐1 BsAb in cell‐based assays. Anti‐tumor activity was confirmed in experimental lung metastasis models and in mice with established subcutaneously transplanted tumors.

**Results:**

The anti‐RANKL/PD‐1 BsAb retained binding to both RANKL and PD‐1 and blocked the interaction with respective counter‐structures RANK and PD‐L1. The inhibitory effect of anti‐RANKL/PD‐1 BsAb was confirmed by demonstrating a complete block of RANKL‐dependent osteoclast formation. Monotherapy activity of anti‐RANKL/PD‐1 BsAb was observed in anti‐PD‐1 resistant tumors and, when combined with anti‐CTLA‐4 mAb, increased anti‐tumor responses. An equivalent or superior anti‐tumor response was observed with the anti‐RANKL/PD‐1 BsAb compared with the combination of parental anti‐RANKL plus anti‐PD‐1 antibodies depending upon the tumor model.

**Discussion:**

Mechanistically, the anti‐tumor activity of anti‐RANKL/PD‐1 BsAb required CD8^+^T cells, host PD‐1 and IFNγ. Targeting RANKL and PD‐1 simultaneously within the tumor microenvironment (TME) improved anti‐tumor efficacy compared with combination of two separate mAbs.

**Conclusion:**

In summary, the bispecific anti‐RANKL/PD‐1 antibody demonstrates potent tumor growth inhibition in settings of ICI resistance and represents a novel modality for clinical development in advanced cancer.

## Introduction

Immunotherapies that target immune checkpoint receptors (e.g. PD‐1 or CTLA‐4) on T cells or PD‐L1 present on tumor and host myeloid cells have shown great advances in the treatment of certain advanced solid organ malignancies.^1^ Importantly, studies in melanoma and NSCLC have demonstrated that anti‐PD‐1/PD‐L1 therapy was more efficacious and less toxic than an antibody targeting CTLA‐4.^2^ However, the overall response rate (ORR) to immunotherapies of these archetypical ‘responsive’ tumor types remains < 50% and a priority now is to improve immunotherapy in order to overcome primary and acquired resistance.^3^, ^4^, ^5^ Combining anti‐CTLA‐4 with anti‐PD‐1 produced superior tumor responses and survival benefit in advanced melanoma, demonstrating the importance of combination strategies which target non‐redundant mechanisms of immune evasion by tumors.^2^ These data demonstrate that simultaneous targeting of complementary immunosuppressive pathways in the tumor microenvironment (TME) may overcome immunotherapy resistance. Novel partners for established immune checkpoint inhibitor (ICI) in the treatment of cancer or novel therapeutic modalities are needed to address the problems of immunotherapy treatment resistance.

RANK (TNFRSF11a) and RANKL (TNFSF11) are members of the tumor necrosis factor receptor and ligand superfamilies, respectively, with closest homology to CD40 and CD40L.^6^ This pathway is currently best known for a role in bone homeostasis, as the differentiation of osteoclasts requires RANKL interaction with RANK expressed on the myeloid osteoclast precursors.^7^ The anti‐RANKL antibody (denosumab) blocks RANKL‐RANK interactions resulting in antagonism of RANK signalling and is widely used in clinical practice as an anti‐resorptive, bone protective agent in patients with bone metastasis or post‐menopausal osteoporosis.^7^ However, despite this clinical focus, the RANKL/RANK pathway was initially described in terms of dendritic cell (DC)–T‐cell biology and RANK signalling in myeloid cells has more recently been recognised to have tolerogenic effects in different contexts^8^, ^9^, ^10^, ^11^ suggesting potential applications of RANKL/RANK antagonism beyond the current, skeletally targeted supportive care applications and, instead, as an anti‐cancer therapy, via immune activation.

Recent preclinical and clinical evidence supports a potential for RANKL/RANK antagonism to enhance anti‐tumor immunity, particularly in combination with ICI.^12^, ^13^ RANK and RANKL are increased in tumors and expressed by various immune cell types in the TME, including RANK by tumor‐infiltrating myeloid cells (TAMCs) and RANKL expression variously by CD8^+^ and CD4^+^ T cells, tumor cells and other stromal components.^7^, ^12^ The combination treatment of anti‐RANKL mAb with immune checkpoint blockade (e.g. mAbs to PD‐1, CTLA‐4 or PD‐L1) consistently enhances control of subcutaneous (s.c.) tumor growth or metastasis across a number of different mouse tumor types (melanoma, prostate, colon, fibrosarcoma and lung), and, importantly, this combination is active in anti‐PD‐1‐resistant settings.^14^, ^15^, ^16^ The addition of anti‐RANKL will also enhance the anti‐tumor efficacy of other immunotherapy strategies, such as vaccination,^16^ or Treg cell depletion.^15^ Moreover, case studies and recent retrospective clinical analyses of patients with advanced melanoma or NSCLC provide ‘real‐world’ clinical evidence that RANKL inhibition may enhance the efficacy of ICI.^17^ The ORRs of bone metastatic NSCLC or melanoma patients upon the addition of anti‐RANKL mAb (denosumab) to ICI appear to be higher than previously reported response rates to ICI monotherapy. Altogether, these data provide preclinical and clinical support that co‐blockade of RANKL and ICI, using two distinct mAbs, targets complementary mechanisms within the TME and improves anti‐tumor efficacy via immune activation.

Bispecific antibody (BsAb) as a modality to target two antigens simultaneously is an emerging strategy to improve clinical efficacy compared with the combination of two separate mAbs.^18^, ^19^ In immuno‐oncology, increased anti‐tumor efficacy and avoidance of resistance may be achieved with BsAbs, compared with the combination of mAb approaches, because of a more complete antagonism of two immunomodulatory pathways simultaneously via avidity effects and a more selective activation of the immune system within the TME. A more tumor‐specific delivery of BsAb resulting from increased target expression within the TME may not only enhance tumor control but also reduce systemic toxicities. The expression of RANK and RANKL within the TME and the potential complementary immunosuppressive function of RANKL/RANK antagonism with ICI, revealed in preclinical and clinical combination studies, indicate that dual targeting of RANKL/RANK and PD‐1/PD‐L1 with a BsAb modality represents a rational therapeutic strategy.

To test this hypothesis, we generated a bifunctional antibody which binds RANKL and PD‐1 simultaneously and characterised *in vitro* activities and efficacy in *in vivo* tumor models. We demonstrate that anti‐RANKL/PD‐1 BsAb is active in controlling lung metastasis and s.c. tumor growth, including responses in tumors which are anti‐PD‐1‐resistant. Moreover, in certain s.c. tumor models, the anti‐RANKL/PD‐1 BsAb was significantly more effective in inhibiting tumor progression than the combination of parental antibodies. Our data demonstrate that a BsAb approach simultaneously blocking RANKL/RANK and the PD‐1/PD‐L1 immune checkpoint in the TME may provide a more effective immunotherapy approach strategy against cancers, including those that fail to respond to current ICI.

## Results

### Design and bifunctional target binding of anti‐RANKL/PD‐1 BsAb)

A anti‐RANKL/PD‐1 BsAb was generated which binds to both muRANKL and muPD‐1 by fusing corresponding Fab‐encoding sequences from anti‐RANKL clone IK22‐5^20^ and anti‐PD‐1 clone RMP1‐14^21^ onto an IgG1 backbone. Assembly of heterodimeric bispecific IgG antibodies was facilitated by engineering of complementary knob‐in‐hole mutations into the CH3 domains of two heavy chains (described in Methods). The desired light‐chain/heavy‐chain pairings were facilitated by an established approach^22^ in which the CH1 and CL sequences of the anti‐PD‐1 RMP1‐14 were interchanged and fused onto the IgG1 Fc; the anti‐RANKL IK22‐5 sequences were unchanged and fused onto IgG1 Fc (Figure 1a). The D265A mutation was also introduced into both chains encoding the IgG1 Fc domain to reduce binding to Fc receptors and reduce effector function. Monospecific controls for both anti‐RANKL and anti‐PD‐1 were generated on the same IgG1 Fc D265A backbones. All recombinant antibodies were produced by transient transfection in mammalian expression system and purified by protein‐A affinity chromatography. Based on SDS‐PAGE and Western blot analysis under non‐reducing conditions, the anti‐RANKL/PD‐1 BsAb was detected with estimated molecular weight of ~ 80 kDa, ~ 100 kDa and 150 kDa (calculated M.W. 145 kDa; Figure 1b). Purity of the anti‐RANKL/PD‐1 BsAb was 85.86%, estimated by SEC‐HPLC (Figure 1c).

**Figure 1:** Design and bifunctional target binding ability of anti‐RANKL/PD‐1 bispecific antibody (BsAb). **(a)** Schematic representation of the structure of anti‐RANKL/PD‐1 BsAb. The anti‐RANKL/PD‐1 BsAb was generated which binds to both muRANKL and muPD‐1 by fusing corresponding Fab‐encoding sequences onto an IgG1 backbone, and heterodimerisation of heavy chains was facilitated as described in Methods. **(b)** The anti‐RANKL/PD‐1 BsAb was produced by transient expression in ExpiCHO‐S suspension cells and purified by protein‐A affinity chromatography. Purified proteins were subsequently analysed by SDS‐PAGE and Western blotting using standard protocols. Purified proteins were either under reducing conditions (lane 1) or under non‐reducing conditions (lane 2). Detection of proteins by Western blotting was performed using goat anti‐human IgG‐HRP. **(c)** SEC‐HPLC analysis of purified anti‐RANKL/PD‐1 BsAb. **(d, e)** The ability of anti‐RANKL/PD‐1 BsAb to block RANK‐Fc or PD‐L1‐Fc was tested in a flow cytometry‐based competition assay in HEK‐293 cells transiently transfected with either **(d)**. muRANKL or **(e)**. muPD‐1. HEK‐293 cells transiently transfected with mouse RANKL or muPD‐1 were incubated with various concentrations of either anti‐RANKL/PD‐1 BsAb (human IgG1 D65A isotype), anti‐RANKL mAb IK22‐5 (rat IgG2a), rat IgG2a isotype control or human IgG1 D65A isotype control. After incubation with biotinylated recombinant mouse RANK‐Fc or mouse PD‐L1‐Fc, bound counter‐structures were detected with streptavidin–APC and analysed by flow cytometry. Representative FACS plots and summary data of inhibition of RANK‐Fc or PD‐L1‐Fc binding of two independent experiments are shown. **(f)** Inhibitory activity of antibodies on osteoclastogenesis *in vitro*. Mouse BM cells cultured in the presence or absence of anti‐IK22‐5 mAb as a positive control, huIgG1 D265A isotype control or anti‐RANKL/PD‐1 BsAb (human IgG1 D65A isotype) at concentrations from 1000 to 50 ng mL^−1^. Culture of BM cells was performed in DMEM supplemented with CSF‐1 and mouse RANKL. Seven days later, TRAP ^+^ multinucleated (more than three nuclei) cells were counted. Data are expressed as means ± SEM of triplicate cultures. Representative TRAP^+^ osteoclast enumeration from three independent experiments is shown.

The ability of the anti‐RANKL/PD‐1 BsAb to block ligand binding was tested in a competition assay with either recombinant muRANK‐Fc or recombinant muPD‐L1‐Fc, the high‐affinity counter‐structures for antibody target antigens. HEK‐293 cells were transiently transfected with either muRANKL or muPD‐1, and binding of the appropriate counter‐structures was measured in a flow cytometry‐based assay. The anti‐RANKL/PD‐1 BsAb was able to fully block RANK‐Fc binding to muRANKL, as did the positive control anti‐RANKL antibody IK22‐5 (Figure 1d). The anti‐RANKL/PD‐1 BsAb demonstrated antagonistic activity in blocking RANK‐Fc binding to RANKL with an IC50 of 2.6 μg mL^−1^, compared an IC50 of 1.1 μg mL^−1^ observed with the control anti‐RANKL mAb IK22‐5. The anti‐RANKL/PD‐1 BsAb also blocked PD‐L1‐Fc binding to PD‐1 (Figure 1e), with a slightly weaker effect to that observed with the control anti‐PD‐1 mAb RMP1‐14. The reduced level of RANKL/RANK‐Fc or PD‐1/PD‐L1‐Fc blocking by anti‐RANKL/PD‐1 BsAb compared with parental (bivalent) antibodies is likely as a result of the monovalent binding nature of the BsAb to each corresponding target antigen. Isotype controls did not affect binding of either RANK‐Fc or PD‐L1‐Fc (Figure 1c, d). The anti‐RANKL/PD‐1 BsAb did not bind untransfected HEK‐293 cells (data not shown).

To evaluate the functional inhibitory effect of the anti‐RANKL/PD‐1 BsAb in a cell‐based functional assay, the effect on *in vitro* osteoclastogenesis was tested. Cells were cultured with CSF‐1 and RANKL for 7 days (with and without antibodies), and then, tartrate‐resistant acid phosphatase (TRAP^+^) multinucleated osteoclast cells were counted. Similar to the effect of the positive control anti‐RANKL antibody IK22‐5, the addition of the anti‐RANKL/PD‐1 BsAb, but not the addition of IgG isotype control, inhibited the formation of TRAP^+^ multinucleated cells in a dose‐dependent manner (Figure 1f). Compared with the parental anti‐RANKL mAb, the anti‐RANKL/PD‐1 BsAb is approximately fivefold to 20‐fold less potent in the *in vitro* osteoclast assay. However, the anti‐RANKL/PD‐1 BsAb demonstrated approximately equivalent inhibitory activity compared with decoy receptor RANK‐Fc control. At a concentration of 250 ng mL^−1^, the anti‐RANKL mAb IK22‐5 and the anti‐RANKL/PD‐1 BsAb both completely blocked osteoclast formation (Figure 1f).

### Efficacy of anti‐RANKL/PD‐1 BsAb in experimental metastasis

In a previous study, we demonstrated that blockade of RANKL with anti‐RANKL mAb (IK22/5) improved anti‐metastatic and anti‐tumor activity achieved with antibodies targeting PD‐1/PD‐L1 in mouse models of melanoma and prostate cancer (Ahern^15^). Here, we aimed to test whether the single‐agent anti‐RANKL/PD‐1 BsAb would at least retain similar efficacy compared to the combination of parental anti‐RANKL plus anti‐PD‐1 antibodies. In wild‐type (WT) mice bearing experimental RM1 prostate cancer lung metastases (Figure 2a) or B16F10 melanoma lung metastases (Figure 2b), combination of the control anti‐RANKL (anti‐RANKL IgG1D265A) and anti‐PD‐1 (anti‐PD‐1 IgG1D265A) antibodies significantly improved metastatic control compared with anti‐PD‐1 treatment alone. Treatment with control anti‐RANKL antibody did not affect RM1 or B16F10 lung metastases. These observations using the newly developed, recombinant forms of anti‐RANKL and anti‐PD‐1 antibodies on IgG1D265A backbone were consistent with the previous study using rat IgG2a hybridoma antibodies.^15^

**Figure 2:** Co‐targeting of RANKL and PD‐1 with bispecific anti‐RANKL/PD‐1 antibody suppresses experimental metastasis to lung. **(a)** Groups of C57BL/6 wild‐type (WT) mice (*n* = 6/group) were injected i.v. with 2 × 10^5^ RM‐1 prostate carcinoma cells. Mice were treated on days −1, 0 and 2 (relative to tumor inoculation) with cIg (200 μg i.p., Mac4 human IgG1 D265A), anti‐RANKL (100 μg i.p., IK22.5 human IgG1 D265A), anti‐PD‐1 (100 μg i.p., RMP1‐14 human IgG1 D265A), combination of anti‐RANKL + anti‐PD‐1 (100 μg i.p. each) and anti‐RANKL/PD‐1 BsAb (100 or 200 μg i.p., human IgG1 D265A) as indicated. Metastatic burden was quantified in the lungs after 14 days by counting colonies on the lung surface. Means ± SEM are shown. **(b)** Groups of C57BL/6 WT mice (*n* = 6–10/group) were injected i.v. with 2 × 10^5^ B16F10 melanoma cells. Mice were treated on days −1, 0 and 2 (relative to tumor inoculation) with cIg (200 μg i.p., Mac4 human IgG1 D265A), anti‐RANKL (100 μg i.p., IK22.5 human IgG1 D265A), anti‐PD‐1 (100 μg i.p., RMP1‐14 human IgG1 D265A), combination of anti‐RANKL + anti‐PD‐1 (100 μg i.p. each) and anti‐RANKL/PD‐1 BsAb (100 or 200 μg i.p., human IgG1 D265A) as indicated. Metastatic burden was quantified in the lungs after 14 days by counting colonies on the lung surface. Means ± SEM are shown. Experiments in **a** and **b** were performed twice. Statistical differences between the indicated groups were determined by one‐way ANOVA and Tukey's multiple comparisons (*P <* *0.05, **P <* *0.01, ***P <* *0.001, ****P <* *0.0001).

In both models, treatment with the anti‐RANKL/PD‐1 BsAb demonstrated a dose‐dependent reduction in lung metastatic burden (data not shown), with the 200 μg BsAb dose treatment resulting in a superior reduction in lung metastases compared with anti‐PD‐1 antibody alone (****P <* *0.0001 for RM1 model; *P <* *0.05 for B16F10 model; Figure 2a, b). Compared with the combination treatments of anti‐PD‐1 plus anti‐RANKL antibodies dosed at 100 μg of each antibody (i.e. 200 μg of total antibody), treatment with the anti‐RANKL/PD‐1 BsAb with an equivalent overall antibody dose (200 μg) achieved at least an equivalent improvement in control of RM1 prostate cancer (Figure 2a) or B16F10 melanoma (Figure 2b) lung metastases. In the RM1 model, a lower treatment dose (100 μg) of anti‐RANKL/PD‐1 BsAb also significantly reduced (***P <* *0.001) lung metastases compared with the combination of anti‐PD‐1 and anti‐RANKL (200 μg of total antibody; Figure 2a).

These data indicate that treatment with the anti‐RANKL/PD‐1 BsAb resulted in significantly greater inhibition of lung metastasis than the anti‐PD‐1 antibody and at least equivalent activity to that achieved with the combination of parental anti‐RANKL plus anti‐PD‐1 antibodies.

### Superior anti‐tumor efficacy of anti‐RANKL/PD‐1 BsAb

The efficacy of the anti‐RANKL/PD‐1 BsAb was next compared with the combination treatment with anti‐RANKL and anti‐PD‐1 antibodies in WT mice bearing s.c. CT26 colon or 3LL lung carcinoma tumors. While both tumor types were unresponsive to anti‐PD‐1 or anti‐RANKL monotherapies, the addition of anti‐RANKL to anti‐PD‐1 significantly suppressed established tumor growth (Figure 3a, b), consistent with the previous report^15^ using rat IgG2a hybridoma antibodies. The 100 and 200 μg doses of the anti‐RANKL/PD‐1 BsAb significantly reduced established s.c. tumor growth of both 3LL and CT26 compared with cIg, anti‐PD‐1 monotherapy or anti‐RANKL monotherapy (****P <* *0.0001 for comparison of BsAb to cIg, anti‐PD‐1 or anti‐RANKL treatment groups in both 3LL and CT26 models). Moreover, treatment with the anti‐RANKL/PD‐1 BsAb (200 μg) significantly improved s.c. tumor control compared with an equivalent overall antibody dose (200 μg) of anti‐RANKL plus anti‐PD‐1 (**P <* *0.01 for both 3LL and CT26 models; Figure 3a, b). Thus, treatment with the single‐agent, anti‐RANKL/PD‐1 BsAb is active in two anti‐PD‐1‐resistant models and demonstrates superior tumor control compared with the combination of individual parental antibodies.

**Figure 3:** Co‐targeting of RANKL and PD‐1 with anti‐RANKL/PD‐1 BsAb suppresses subcutaneous tumor growth. **(a)** Groups of C57BL/6 WT mice (*n* = 6–10/group) were injected s.c. with 5 × 10^5^ 3LL lung carcinoma cells. Mice were treated on days 8, 12, 16 and 20 post‐tumor inoculation with cIg (200 μg i.p., Mac4 human IgG1 D265A), anti‐RANKL (100 μg i.p., IK22.5 human IgG1 D265A), anti‐PD‐1 (100 μg i.p., RMP1‐14 human IgG1 D265A), combination of anti‐RANKL + anti‐PD‐1 (100 μg i.p. each) and anti‐RANKL/PD‐1 BsAb (100 or 200 μg i.p., human IgG1 D265A) as indicated. Tumor area (mm^2^) was measured every 2–4 days, and means ± SEM are shown. **(b)** Groups of BALB/c WT mice (*n* = 6or7/group) were injected s.c. with 1 × 10^5^ CT26 colon adenocarcinoma cells. Mice were treated on days 9, 13, 17 and 21 (relative to tumor inoculation) with cIg (200 μg i.p., Mac4 human IgG1 D265A), anti‐RANKL (100 μg i.p., IK22.5 human IgG1 D265A), anti‐PD‐1 (100 μg i.p., RMP1‐14 human IgG1 D265A), anti‐RANKL + anti‐PD‐1 (100 μg i.p. each) and anti‐RANKL/PD‐1 BsAb (100 or 200 μg i.p., human IgG1 D265A) as indicated. Tumor area (mm^2^) was measured every 2–4 days, and means ± SEM are shown. The experiment was performed once. Statistical differences between the indicated groups were determined by two‐way ANOVA with Tukey's post‐test analysis (*P <* *0.05, **P <* *0.01, ****P <* *0.0001). The arrow indicates the day that therapy was initiated.

### Anti‐tumor efficacy of anti‐RANKL/PD‐1 BsAb is dependent on CD8^+^ T cells, host PD‐1 and IFNγ

In order to address mechanisms by which the anti‐RANKL/PD‐1 BsAb controls tumor growth, we examined whether the efficacy was dependent on IFNγ or CD8^+^ T cells in the more immunogenic MC38‐OVA^dim^ colon adenocarcinoma model. Similar to the response to combination of anti‐RANKL plus anti‐PD‐1 antibodies, treatment with either 100 or 200 μg of the anti‐RANKL/PD‐1 BsAb significantly controlled established MC38‐OVA^dim^ colon tumor growth compared with anti‐PD‐1 monotherapy (****P <* *0.0001; Figure 4a). Importantly, treatment with 200 μg of anti‐RANKL/PD‐1 BsAb significantly improved the tumor rejection rate (12/15 mice) vs. combination of anti‐RANKL plus anti‐PD‐1 antibodies (3/15; Fisher's exact test **P =* *0.0028). No mice rejected MC38‐OVA^dim^ s.c. tumors (0/15) after treatment with cIg or anti‐RANKL antibody, while treatment with anti‐PD‐1 antibody alone resulted in few tumor rejections (1/15).

**Figure 4:** Anti‐RANKL/PD‐1 BsAb suppresses MC38‐OVA ^dim^ colon adenocarcinoma growth in CD8^+^T‐cell‐ and IFNγ‐dependent manner. **(a)** Groups of C57BL/6 wild‐type (WT) mice (*n* = 10/group) were injected s.c. with 1 × 10^6^ MC38‐OVA ^dim^ colon adenocarcinoma cells. Mice were treated on days 12, 16, 20 and 24 (relative to tumor inoculation) with cIg (200 μg i.p., Mac4 human IgG1 D265A), anti‐RANKL (100 μg i.p., IK22.5 human IgG1 D265A), anti‐PD‐1 (100 μg i.p., RMP1‐14 human IgG1 D265A), anti‐RANKL + anti‐PD‐1 (100 μg i.p. each) and anti‐RANKL/PD‐1 BsAb (100 or 200 μg i.p., human IgG1 D265A) as indicated. Tumor area (mm^2^) was measured every 2–4 days, and means ± SEM are shown. **(b)** Groups of C57BL/6 wild‐type (WT) mice (*n* = 10/group) were injected s.c. with 1 × 10^6^ MC38‐OVA ^dim^ colon adenocarcinoma cells. Mice were treated on days 12, 16, 20 and 24 (relative to tumor inoculation) with cIg (200 μg i.p., Mac4 human IgG1 D265A) or anti‐RANKL/PD‐1 BsAb (200 μg i.p., human IgG1 D265A) as indicated. Some groups of mice were treated with either cIg (100 μg), anti‐CD8β (100 μg) or anti‐mIFNγ (250 μg) on days 11, 12 and 19, relative to tumor inoculation. Tumor area (mm^2^) was measured every 2–4 days, and means ± SEM are shown. Experiment was performed once. Statistical differences between the indicated groups were determined by two‐way ANOVA and Tukey's multiple comparisons (*P <* *0.05, ** *P *<* *0.01, **** *P *<* *0.0001). The arrow indicates the day that therapy was initiated.

Given that the MC38‐OVA^dim^ s.c. model thus represented a setting in which anti‐RANKL/PD‐1 demonstrated superior tumor control vs. combination of parental anti‐RANKL plus anti‐PD‐1 antibodies, we investigated the mechanisms related to this efficacy. In WT mice bearing MC38‐OVA^dim^ tumors, CD8^+^ T cells and IFNγ were critical for the efficacy of the anti‐RANKL/PD‐1 BsAb therapy as depletion of CD8^+^ T cells or neutralisation of IFNγ in these treated mice abrogated the anti‐tumor response (Figure 4b).

To address the contribution of host PD‐1 towards anti‐RANKL/PD‐1 BsAb efficacy, we utilised the AT3‐OVA^dim^ breast adenocarcinoma model that is non‐responsive to anti‐PD‐1^23^ in WT mice. Similar to responses observed in other s.c. tumor models, treatment with the anti‐RANKL/PD‐1 BsAb (100 or 200 μg) or combination of anti‐RANKL plus anti‐PD‐1 antibodies significantly controlled AT3‐OVA^dim^ established tumor growth in WT mice compared with anti‐PD‐1 monotherapy (****P <* *0.0001; Figure 5). In contrast to activity in WT mice, efficacy of anti‐RANKL/PD‐1 BsAb on AT3‐OVA^dim^ tumor growth was negated in *Pdcd1* ^*−/−*^ mice (Figure 5), indicating the requirement for host PD‐1.

**Figure 5:** Anti‐RANKL/PD‐1 BsAb suppresses subcutaneous AT3‐OVA ^dim^ tumor growth in a PD‐1‐dependent manner. Groups of C57BL/6 WT or *Pdcd1* ^−/−^ mice (*n* = 5–6/group) were injected s.c. with 1 × 10^6^ AT3‐OVA ^dim^ on day 0, and tumor growth was monitored. Mice were treated i.p. on days 20, 24, 28 and 31 (relative to tumor inoculation) with the following antibodies: cIg (recombinant MAC4 huIgG1 D265A; 200 μg), anti‐RANKL/PD‐1 BsAb (huIgG1 D265A; 100 μg or 200 μg, as indicated), anti‐PD‐1 (recombinant RMP1‐14 huIgG1 D265A; 100 μg), anti‐RANKL (recombinant IK22‐5 huIgG1 D265A; 100 μg) or their combinations as indicated. Tumor area (mm^2^) was measured every 2–4 days, and means ± SEM are shown. Experiment was performed once. Statistical differences between the indicated groups were determined by two‐way ANOVA and Tukey's multiple comparisons (****P <* *0.0001). The arrow indicates the day that therapy was initiated.

### Anti‐RANKL/PD‐1 BsAb enhances the anti‐tumor efficacy of anti‐CTLA‐4 treatment

Given that combination immune checkpoint blockade of CTLA‐4 and PD‐1 provides a superior clinical benefit compared with either monotherapy treatment alone in certain patient groups^2^ and is emerging as standard of care, we next compared the efficacy of anti‐RANKL/PD‐1 BsAb to combination of anti‐PD‐1 plus anti‐CTLA‐4 therapies. As shown previously (Figure 3b), neither anti‐RANKL nor anti‐PD‐1 antibodies (100 μg) had significant effects as monotherapies in CT26 tumor‐bearing mice. Significant suppression of established tumor growth was observed with anti‐CTLA‐4 monotherapy treatment (****P <* *0.0001 compared to cIg; Figure 6). The addition of anti‐PD‐1 antibody to anti‐CTLA‐4 antibody resulted in superior tumor control than treatment with anti‐CTLA‐4 monotherapy (****P <* *0.0001; Figure 6), consistent with the superior efficacy of combination treatment vs. monotherapy in advanced cancer patients.^2^ Treatment of mice with established CT26 tumors with the anti‐RANKL/PD‐1 BsAb resulted in a significantly greater response compared with anti‐CTLA‐4 monotherapy (****P <* *0.0001) and an equivalent tumor control compared with the combination of anti‐PD‐1 plus anti‐CTLA‐4 antibodies (n.s. difference between groups; Figure 6).

**Figure 6:** Anti‐RANKL/PD‐1 BsAb enhances the anti‐tumor efficacy of anti‐CTLA‐4 in the CT26 tumor model. Groups of BALB/c mice (*n* = 5–17/group) were injected s.c. with 1 × 10^5^ CT26 on day 0, and tumor growth was monitored. Mice were treated i.p. on days 9, 17, 18 and 21, relative to tumor inoculation, with the following antibodies: cIg (to a total of 300 μg), anti‐RANKL/PD‐1 BsAb (huIgG1D265A backbone; 200 μg), anti‐CTLA4 (UC10‐4F10, 100 μg), anti‐PD‐1 (RMP1‐14, 100 μg), anti‐RANKL (IK22‐5, 100 μg) or their combinations as indicated. Tumor area (mm^2^) was measured every 2–4 days, and means ± SEM are shown. The experiment was performed once. Statistical differences between the indicated groups were determined by two‐way ANOVA and Tukey's multiple comparisons (****P <* *0.0001). The arrow indicates the day that therapy was initiated.

We next assessed whether the addition of anti‐RANKL/PD‐1 BsAb could further improve the anti‐tumor efficacy of combined anti‐CTLA‐4 and anti‐PD‐1 therapy. The triple combination of anti‐PD‐1, anti‐RANKL and anti‐CTLA‐4 antibodies was more efficacious in suppression of CT26 s.c. growth than with any dual therapy, consistent with our previous report using hybridoma mAbs.^15^ Similarly, the addition of anti‐RANKL/PD‐1 BsAb to anti‐CTLA4 suppressed tumor growth of CT26 tumor‐bearing mice and resulted in a significantly greater anti‐tumor efficacy than any dual combination therapy tested (Figure 6).

## Discussion

In this study, we report that the concurrent neutralisation of RANKL and PD‐1 by a BsAb consistently demonstrated superior anti‐tumor or anti‐metastatic control to monotherapies, even in settings in which anti‐PD‐1 or anti‐CTLA‐4 treatment alone evoked minimal anti‐tumor activities. Moreover, treatment with the anti‐RANKL/PD‐1 BsAb achieved superior anti‐tumor control compared with the combination of anti‐RANKL plus anti‐PD‐1 in multiple s.c. tumor models and demonstrated equivalent anti‐tumor control to the currently most effective immunotherapy combination (anti‐PD‐1 plus anti‐CTLA‐4).

The superior efficacy of anti‐RANKL/PD‐1 BsAb could be a consequence of simultaneously blocking two non‐redundant, immunosuppressive pathways in the TME. In our study, depletion of CD8^+^ T cells or neutralisation of IFNγ abrogated the anti‐tumor efficacy of anti‐RANKL/PD‐1 BsAb suggesting major roles for adaptive immune cells in the response. The key contribution of CD8^+^ T cells and IFNγ as a mechanism for increased anti‐tumor immunity upon PD‐1 blockade is well established^1^ and is likely to be mechanistically linked to anti‐RANKL/PD‐1 BsAb efficacy. The mechanistic contribution of RANKL/RANK blockade towards anti‐RANKL/PD‐1 BsAb efficacy may be informed by previously published data in which anti‐RANKL mAb added to ICI resulted in increased CD8^+^ T‐cell infiltrates in tumors and increased Th1‐type cytokine production (e.g. IFNγ, IL‐2) by TILs compared with ICI alone.^14^, ^15^ The additive contributions of RANKL/RANK blockade to ICI, potentially via interruption of an immunosuppressive myeloid–lymphocyte axis and/or cross‐modulation of RANKL/RANK and PD‐1/PD‐L1 expression within the TME as described in earlier studies,^14^, ^15^ would also factor into the mechanism by which anti‐RANKL/PD‐1 BsAb enhances anti‐tumor immunity and controls tumor growth.

While thymic expression of RANKL and RANK and the potential role for this pathway in negative selection may contribute to some aspects of combination efficacy of RANK/RANKL antagonism with ICI,^16^, ^24^ the observed distribution of RANK and RANKL within the TME more likely informs the distinct mechanisms by which the anti‐RANKL/PD‐1 BsAb evokes superior anti‐tumor immunity and efficacy. Approximately 20% of TILs in mouse tumors expressed RANK with greater than 90% also positive for CD11b, suggesting intratumor RANK was expressed almost exclusively by TAMCs, which includes tumor‐associated macrophages (TAM), myeloid‐derived suppressor cells and DC.^14^, ^15^ RANK expression on CD11b+ TAMs is associated with CD206 but low MHCII expression, indicative of immunosuppressive M2‐type TAMs.^14^ These findings are consistent with observations in human tumors, where RANK expression is frequently co‐localised with the macrophage markers CD163, arginase‐1 (Arg1), and CD206^10^, ^11^ and tolerogenic function.^9^, ^10^, ^11^

However, RANKL has been reported to be expressed at a generally low frequency overall in mouse TILs (on < 10% of infiltrating T cells, including Ki67+/antigen‐experienced T cells), with a higher proportion of CD8^+^ than CD4^+^ T cells expressing RANKL.^14^ Relevant to the mechanism of the anti‐RANKL/PD‐1 BsAb, previous expression analysis in mouse tumors has demonstrated that almost all CD8^+^RANKL^+^ T‐cell TILs (> 90%) co‐expressed PD‐1; in comparison, <40% CD8^+^RANKL^−^ T‐cell TILs were PD‐1‐positive.^15^ Alternatively, the immunosuppressive RANKL signal may originate from certain lymph node stromal cells [marginal reticular cells (MRCs)],^25^ tumor cells themselves,^26^ NK cells or ILC3s.^27^

Together, these findings support the hypothesis that RANKL, originating from various sources, mediates RANK signalling in TAMCs and immunosuppressive/tolerogenic effects in the TME. The inhibition of immunosuppressive TAMCs and increased TIL infiltration achieved by RANKL/RANK blockade complements the reversal of CD8^+^ T‐cell dysfunction resulting from PD‐1 blockade, leading to an enhanced anti‐tumor effect. The superior anti‐tumor efficacy of anti‐RANKL/PD‐1 BsAb compared with the combination of anti‐RANKL plus anti‐PD‐1 antibodies may be explained by an enriched biodistribution of the BsAb to elevated levels of RANKL and PD‐1 expressed in the TME, including, but not limited to, co‐expression of both target antigens on CD8^+^ TILs. The resulting avidity increase achieved by co‐targeting two antigens simultaneously may result in a more tumor‐selective targeting and greater blockade of immunosuppressive pathways. Both denosumab (anti‐RANKL) and anti‐PD‐1/PD‐L1 mAbs result in some systemic toxicities as monotherapies.^28^, ^29^ However, whether the more tumor‐selective biodistribution of anti‐RANKL/PD‐1 BsAb mitigates any toxicities resulting from either monotherapy or combination of anti‐RANKL plus anti‐PD‐1/PD‐L1 antibodies remains to be tested.

In general, challenges to the development of BsAbs and future clinical testing potentially include the necessity of additional tailoring of patient stratification markers to each binding arm of the BsAb, or the unique combinatorial biology elicited as a result of simultaneously targeting two pathways in the TME. Ongoing work to more comprehensively define the distribution of RANK and RANKL in human tumors and the precise cell target and mechanism by which RANKL blockade enhances ICI efficacy and anti‐tumor immunity are critical. These data are necessary to identify potential patient stratification and pharmacodynamic biomarkers to guide application of a novel anti‐RANKL/PD‐1 BsAb modality in oncology.

The discovery of immune checkpoints and subsequent clinical development of ICIs, particularly mAbs targeting PD‐1, have revolutionised the field of oncology, providing patients with difficult‐to‐treat cancers much needed immunotherapy options. However, broader application of current ICIs, including anti‐PD‐1, anti‐PD‐L1 and anti‐CTLA‐4 mAbs, is limited by primary or acquired resistance such that only a fraction of cancer patients shows durable benefit. The current study identifies a new bispecific modality that simultaneously inhibits PD‐1/PD‐L1 and RANK/RANKL in the TME, providing benefit in ICI‐resistant settings and demonstrating superior anti‐tumor control compared with the combination of parental anti‐RANKL plus anti‐PD‐1 antibodies. The utility and practicality of the anti‐RANKL/PD‐1 BsAb strategy is illustrated not only by BsAb monotherapy activity in anti‐PD‐1‐resistant models, but also by the ability of anti‐RANKL/PD‐1 BsAb to combine with anti‐CTLA‐4 blockade, further enhancing anti‐tumor efficacy. These results encourage additional preclinical and mechanistic testing as well as clinical development of novel BsAb modalities that simultaneously target RANKL/RANK and PD‐1/PD‐L1 in cancer.

## Methods

### Antibodies and other protein reagents

In order to construct recombinant monospecific anti‐RANKL, monospecific anti‐PD‐1, bispecific anti‐RANKL/PD‐1 and isotype control (MAC4) antibodies, the mAb cDNA sequences were obtained from rat IgG2a hybridomas encoding anti‐RANKL IK22‐5,^20^ MAC4 and anti‐PD‐1 RMP1‐14.^21^ The MAC4 antibody is reactive with anti‐glycoprotein of Chlamydomonas reinhardtii and is therefore a non‐reactive isotype control for *in vitro* and *in vivo* experiments. Sequence analysis of immunoglobulin variable regions and determination of framework and CDRs were achieved using NCBI Nucleotide BLAST, IMGT/V Quest program and NCBI IgBLAST algorithms. For the construction of recombinant monospecific and bispecific antibodies, the rat VH and VL antibody sequences were each fused to human IgG1 Fc sequences with either the ‘knob’ mutation (T366W) introduced into the CH3 domain or three ‘hole’ mutations (T366S, L368A and Y407V) were introduced into the complementary heavy chain. In addition, two Cys residues were introduced (S354C on the ‘knob’ and Y349C on the ‘hole’ side) in order to form a stabilising disulphide bridge and further enhance heterodimerisation. Furthermore, a D265A mutation was also introduced into all IgG1 Fc chains, to abrogate effector function of resulting antibody.

For the construction of recombinant anti‐RANKL/PD‐1 BsAb, the association of the desired light‐chain/heavy‐chain pairings within the heterodimeric BsAb was promoted by the ‘CrossMabVH‐VL’ approach.^30^ Specifically, the RMP1‐14 (anti‐PD‐1 antibody) sequence was engineered as a ‘CrossMabCH1‐CL’, in which the CH1 and CL sequences were interchanged (termed RMP1‐14 CH‐CL‐ huIgG1Fc). The Fab region of the anti‐RANKL antibody (IK22‐5) was unchanged (termed IK22‐5‐huIgG1Fc WT). In order to produce recombinant antibodies, cDNAs encoding each of the appropriate four chains were subcloned into the mammalian expression vector pcDNA3.4 and transfection grade plasmids were maxi‐prepared according to standard techniques. Antibodies were produced by transient expression in ExpiCHO‐S suspension cells grown in serum‐free ExpiCHO Expression Medium (Thermo Fisher Scientific, Waltham, MA, USA) with four expression plasmids (encoding heavy and light chains for different constructs) at equimolar ratios. The cells (1L culture volume) were maintained in Erlenmeyer flasks (Corning Inc., Corning, NY, USA) at 37°C with 8% CO_2_ on an orbital shaker, and the cell culture supernatant collected on day 14 post‐transfection was used for purification. Antibody titres were in the range of transient expression titres of conventional IgG1 antibodies. Cell culture broth was centrifuged followed by filtration. Filtered supernatant was loaded onto a Monofinity A Resin Prepacked Column 1 mL (GenScript, Piscataway, NJ, USA) at 1.0 mL min^−1^. After washing and elution with appropriate buffers, the eluted fractions of the antibody were pooled and buffer exchanged to PBS, pH 7.2. Protein was sterilised via a 0.22‐μm filter, packaged aseptically and stored at −80°C.

Purified anti‐mouse anti‐RANKL (IK22/5; rat IgG2a), anti‐CTLA‐4 (UC10‐4F10, hamster IgG) and control antibodies (cIg; hamster cIg, or 1–1 or 2A3, rat IgG2a) were purchased from BioXcell (West Lebanon, NH, USA). Anti‐PD1 clone RMP1‐14 (rat IgG2a) was purchased from Leinco (St Louis, MO, USA). Antibodies to deplete CD8 T cells (53.5.8; BioXcell) and neutralising IFNγ (H22; Leinco) were administered at the dose and schedule as indicated in the Figure captions.

Production of recombinant mouse RANK‐Fc was as follows. The cDNA sequences encoding mouse RANK sequence (AA 31–214), the linker IEGRDID and human IgG1 Fc sequence (AA100‐Lys330) were subcloned into the mammalian expression vector pcDNA3.4. Protein was produced after transient transfection of Expi293F cells, and protein was obtained from supernatant of cell culture followed by a one‐step purification by Monofinity A Resin Prepacked Column. Purity of protein was estimated to be 85%, based on densitometric analysis of the Coomassie Blue‐stained SDS‐PAGE gel under non‐reducing conditions and SEC‐HPLC. Recombinant muPD‐L1‐Fc produced and purified from HEK‐293 cells was purchased from Sino Biological (Wayne, PA, USA).

### cDNAs

pCMV3‐mTNFSF11 and pCMV3‐mPDCD1 plasmid constructs were obtained from Sino Biological Inc.

### Cell culture

B16F10 mouse melanoma (ATCC, Manassas, VA, USA), prostate carcinoma RM‐1 (ATCC; Pam Russell, University of Sydney, 1996), colon carcinoma CT26 (Robert Wiltrout, National Cancer Institute Frederick, 1991), colon carcinoma MC38‐OVA^dim,^ 31 3LL Lewis triple lung carcinoma (Dr Michael Holzel, University of Bonn, 2019) and AT3‐OVA^dim^ mammary carcinoma^32^ were obtained and injected as previously described.^33^ All the cell lines were maintained in culture for no more than 7 days and were routinely tested for *Mycoplasma* but cell line authentication was not routinely performed.

### Mice

C57BL/6 or BALB/c WT mice were bred‐in‐house at QIMR Berghofer Medical Research or purchased from the Walter and Eliza Hall Institute for Medical Research, Parkville, Victoria, Australia. *Pdcd1* ^*−/−*^ mice^34^ were kindly provided by Michelle Wykes (QIMR Berghofer). All mice were bred and maintained at QIMR Berghofer Medical Research Institute. Eight‐ to twelve‐week‐old mice were used for tumor challenge experiments. Groups of 6–10 mice per experiment were used for both experimental lung metastases and subcutaneous tumor growth assays. All experiments were approved by the QIMR Berghofer Medical Research Institute Animal Ethics Committee.

### Subcutaneous tumor models

For 3LL (5 × 10^5^), CT26 (1 × 10^5^), AT3‐OVA^dim^ (1 × 10^6^) and MC38‐OVA^dim^ (1 × 10^6^) tumor formation, cells were inoculated s.c. into the abdominal flank of WT mice. In the case of AT3‐OVA^dim^, *Pdcd1* ^*−/−*^ gene‐targeted mice were also used. Therapeutic antibody treatment commenced as indicated on day 8–20 after tumor inoculation and was given every 3–4 days for four doses. Additionally, where indicated, anti‐CD8β or anti‐IFNγ antibodies were administered on days 11, 12 and 19, relative to tumor inoculation. Digital callipers were used to measure the perpendicular diameters of the tumors. Tumor sizes were determined by calliper square measurements of two perpendicular diameters with data represented as mean ± SEM (mm^2^) for each group.

### Experimental lung metastasis models

Single‐cell suspensions of B16F10 (2 × 10^5^) or RM‐1 (2 × 10^5^) were injected i.v. into the lateral tail vein of C57BL/6 WT mice. Lungs were harvested on day 14, and surface tumor nodules were counted under a dissection microscope. Antibody treatments were as indicated, with therapeutic antibodies administered on days −1, 0 and 2, relative to tumor inoculation.

### *In vitro* osteoclastogenesis assay

The methods for the *in vitro* TRAP^+^ osteoclast assays were essentially as described.^35^ Bone marrow cells were obtained from two femurs of 8‐week‐old male C57BL/6 WT mice, processed and plated on a 96‐well plate at a density of 2 × 10^4^ cells per plate, in 200 μL per well of complete DMEM with 10% foetal calf serum and 50 ng mL^−1^ of human recombinant CSF‐1 (R&D Systems, Minneapolis, MN, USA). After 48 h at 37°C, media were replenished with complete DMEM, 50 ng mL^−1^ human recombinant CSF‐1 plus 200 ng mL^−1^ of soluble mouse RANKL (Miltenyi Biotec, Auburn, CA, USA) and various concentrations in a serial dilution fashion of either anti‐RANKL mAb (IK22.5 rat IgG2a), anti‐RANKL/PD‐1 BsAb (human IgG1 D265A) or isotype control (human IgG1 Fc). Media and appropriate reagents were replenished every 48 h, and after 7 days, cells were *in situ* stained with TRAP and TRAP^+^ multinucleated (more than three nuclei) cells were enumerated under the pathology microscope.

### RANK‐ and PD‐L1‐blocking ability of anti‐RANKL/PD‐1 BsAb

The ability of the anti‐RANKL/PD‐1 BsAb to block ligand binding was tested in a competition assay with either recombinant muRANK‐Fc or recombinant PD‐L1‐Fc. Recombinant proteins were biotinylated using EZ‐Link Sulfo‐NHS‐LC‐LC Biotin from Thermo Fisher Scientific essentially as described.^36^ Single‐cell suspensions of HEK‐293 were transiently transfected by either the mouse RANKL or mouse PD‐1 using standard FuGENE^®^ 6 (Promega, Madison, WI, USA) transfection procedures. Analysis of RANK‐Fc or PD‐L1‐Fc and competition by antibodies were analysed using a three‐step incubation procedure by flow cytometry 48 h post‐transfection. Samples were firstly incubated with various concentrations in a serial dilution manner of anti‐RANKL (IK22.5; rat IgG2a (BioXcell), anti‐RANKL (human IgG1 D265A), anti‐PD‐1 (human IgG1 D265A), anti‐RANKL/PD‐1 BsAb (human IgG1 D265A), isotype control (1–1; rat IgG2a; BioXcell) or isotype control (human IgG1 D265A) for 30 min on ice. Next, cells were incubated with 2.5 μg of biotinylated murine RANK‐Fc protein or murine PD‐L1‐Fc for an additional 30 min on ice followed by a final incubation with goat anti‐human secondary antibody AF‐647 or streptavidin 1/100 dilution for 30 min on ice. All samples were acquired, and all data were collected on FACSCanto II (BD, Franklin Lakes, NJ, USA) flow cytometer and analysed with FlowJo v10 software (Tree Star, Inc., Ashland, OR, USA).

### Statistical analyses

Statistical analyses were determined with GraphPad Prism 7 (GraphPad Software, San Diego, CA, USA). Significance of differences was calculated by two‐way ANOVA as necessary. Tukey's multiple comparisons tests were utilised unless otherwise indicated. Differences between two groups are shown as the mean ± SD or the mean ± SEM. Data were considered to be statistically significant where the *P* value was equal to or less than 0.05.
